# Protective effect of autophagy on endoplasmic reticulum stress induced apoptosis of alveolar epithelial cells in rat models of COPD

**DOI:** 10.1042/BSR20170803

**Published:** 2017-11-15

**Authors:** Yao Tang, Qi-Hang Cai, Yong-Jian Wang, Shao-Hua Fan, Zi-Feng Zhang, Meng-Qi Xiao, Jin-Yu Zhu, Dong-Mei Wu, Jun Lu, Yuan-Lin Zheng

**Affiliations:** 1 Key Laboratory for Biotechnology on Medicinal Plants of Jiangsu Province, School of Life Science, Jiangsu Normal University, Xuzhou 221116, P.R. China; 2 Department of Respiration, Huaihe Hospital of Henan University, Kaifeng 475000, P.R. China

**Keywords:** Chronic obstructive pulmonary disease, Endoplasmic reticulum stress, Alveolar epithelial cells, Autophagy, Apoptosis

## Abstract

During the present study, we explored the protective effects of autophagy on endoplasmic reticulum (ER) stress (ERS) induced apoptosis belonging to alveolar epithelial cells (AECs) in rat models with chronic obstructive pulmonary disease (COPD). Fifty-six 12-week-old male Sprague–Dawley (SD) rats were randomly assigned into the COPD group (rats exposed to cigarette smoke (CS)), the 3-methyladenine (3-MA) intervention group (COPD rats were administrated with 10 mg/kg autophagy inhibitors), the chloroquine (CQ)-intervention group (COPD rats were administrated 40 mg/kg CQ), and the control group (rats breathed in normal saline). The forced expiratory volume in 0.3 s/forced vital capacity (FEV_0.3_/FVC%), inspiratory resistance (RI), and dynamic lung compliance (Cdyn) were measured and recorded. The expressions of PKR-like ER kinase (PERK) and CCAAT/enhancer-binding protein-homologous protein (CHOP) were detected by immunohistochemistry. The cell apoptotic rates of AECs were analyzed by terminal deoxynucleotidyl transferase (TdT) mediated dUTP-biotin nick end-labeling (TUNEL) staining. The expression levels of light chain 3 (LC3-II), p62, Beclin-1, ATG5, ATG7, Caspase-12, and Caspase-3 were detected by Western blotting. Results showed that the COPD group exhibited a lower FEV_0.3_/FVC% and Cdyn, and a higher RI than the control group. Compared with the control group, the integrated optical density (IOD) values of PERK and CHOP, the apoptotic rate of AECs, and expressions of LC3-II, Beclin-1, ATG5, ATG7, Caspase-3, and Caspase-12 expressions were significantly higher, whereas p62 expression was significantly lower in the COPD group. Based on the results obtained during the present study, it became clear that the inhibition of autophagy could attenuate the ERS-induced apoptosis of AECs in rats with COPD.

## Introduction

Chronic obstructive pulmonary disease (COPD) is a term used to describe a group of diseases that previously included bronchitis and emphysema [1]. COPR is characterized as a progressive disease that generally manifests itself with persistent airflow limitation and enhanced chronic inflammatory response in the lung tissues [2]. The global initiative for COPD (GOLD) has defined COPD as “a common preventable and treatable disease characterized by persistent airflow limitation that is usually progressive and associated with an enhanced chronic inflammatory response in the airways and the lung to noxious particles or gases. Exacerbations and comorbidities contribute to the overall severity in individual patient.” COPD is reported as the dominating cause of death, and the estimated worldwide prevalence is up to 10.1% with a growing tendency in the next few decades [3]. COPD is more common in the older population and is highly prevalent in those aged more than 75 years. The global prevalence of COPD in adults that are older than 40 years is approximately 9–10% [4]. Long-term exposure to cigarette smoke (CS) is the principal and primary risk factor of COPD that accounts for more than 90% of cases [5]. Of those who smoke, approximately 20% will get COPD, and those who have been smoking for their lifetime, 50% will get COPD [6]. Additionally, age, sex, tuberculosis, and exposure to biomass fuels also are important factors associated with COPD [7,8]. Moreover, Płusa [9] verified a critical role of genetic factors in the morbidity of COPD. The morbidity of COPD is slightly higher in male patients than in female patients, five times higher in heavy smokers than in non-smokers, and two times higher in patients with a chronic cough than in asymptomatic patients [10]. Emphysema has been identified as one of the main pathophysiological features that are present during COPD. It is characterized by an expanded alveolar space, depressed lung function, devastated alveolar wall, increased inflammatory cells, and leads to increased cell apoptosis in rats [11,12]. The destruction of connective tissue of the lungs leads to emphysema, which ultimately leads to poor airflow, poor absorption, and release of respiratory gases [2]. Interestingly, endoplasmic reticulum (ER) stress (ERS) has been found to play a role in emphysema and induces apoptosis of alveolar epithelial cells (AECs) subsequently causing lung fibrosis [13].

ER is a unique organelle for protein synthesis, folding, and delivery in the cell and it is essential in numerous cellular functions [14]. An imbalanced calcium status caused by noxious stimuli such as drugs, free radicals, disturbance of calcium metabolism, and hypoxia or an elevated content of unfolded or misfolded proteins in the ER lumen can lead to ERS [15,16]. CS inhalation has been found to induce ERS in rats with COPD, subsequently resulting in lung injury, which might be an original target for protecting AECs from ERS injury in emphysema [17]. The activation of the signaling pathway involving ERS-associated apoptosis is possibly achieved by the increased levels of cleaved Caspase-12 and CCAAT/enhancer-binding protein-homologous protein (CHOP) [18]. Ryter et al. [19] reported that the activation of autophagy in COPD lung specimens was correlated with an increase in epithelial cell apoptosis subjected to CS exposure. Thus, in our experiment, we created rat models of COPD by exposing them to CS in order to explore the effects of autophagy on the ERS-induced apoptosis of AECs in COPD.

## Materials and methods

### Animal grouping and model establishment

A total of 56 specific pathogen-free (SPF) male Sprague–Dawley (SD) rats that were 12 weeks old and weighed between 250 and 280 g were used in the present study. Rats were initially allowed to acclimate for 1 week. All the rats were randomly assigned and evenly divided into four experimental groups with 14 rats in each group: the control group, the COPD group, the chloroquine (CQ) intervention group, and the 3-methyladenine (3-MA; an inhibitor of autophagy) intervention group. Rats in the COPD group were anesthetized on the 1st and the 14th day, and an incision was made to expose the trachea for intratracheal instillation of lipopolysaccharide (LPS; 200 μg/200 μl; Sigma–Aldrich Chemical Company, St. Louis, MO, U.S.A.) using a 4-gauge needle. Rats were then exposed to CS produced by 12 filter-tipped Furongwang cigarettes obtained from the Cigarette Factory (Changde, Hunan). Exposure to CS was performed in a 72-l closed glass box for 0.5 h everyday, starting from the 2nd to the 13^th^ day and from the 15th to the 28th day. Rats in the 3-MA intervention group were used to establish the rat model of COPD, and were intraperitoneally injected with 3-MA (10 mg/kg), 0.5 h before exposure to CS and intratracheal instillation of LPS. Rats in the CQ intervention group were intraperitoneally injected with 3-MA (40 mg/kg), 0.5 h before exposure to CS and intratracheal instillation of LPS except for preparing the COPD model. Rats in the control group received intratracheal instillation of sterilized normal saline on the 1st and the 14th day. From the 2nd to the 13th day and from the 15th to the 28th day, rats were left to breathe in a glass box with normal air for the same period of time with rats in the other groups. General conditions and statuses of all rats were observed everyday, including their diet, activities, cough, and other general conditions, and they were fed a normal diet for 4 weeks before further experiments.

### Pulmonary function testing

Anesthetized rats in each group were positioned in the supine position on the operation table, and an incision was made in the anterior part of the neck in order to expose the trachea and insert a tracheal intubation tube. The other end of tracheal intubation was connected to a pressure sensor, a flow sensor, a ventilator, and Maclab data acquisition system (Buxco Electronics Inc., Troy, NY, U.S.A.). The tidal volume was set at 10 ml/kg, and the respiratory rate was set at 60 breaths/min. The breathing pattern of the rats was observed for a period of time, after which air was rapidly inflated into the trachea with a volume of five times the tidal volume. The ventilator was then immediately disassembled and replaced with an aspirator of negative pressure for air removal. Afterward, the forced expiratory volume in 0.3 s/forced vital capacity (FEV_0.3_/FVC%), inspiratory resistance (RI), and dynamic lung compliance (Cdyn) were calculated by Maclab data acquisition system.

### Lung tissue collection

Rats were intraperitoneally anesthetized with 2% pentobarbital sodium in a sterile environment (20 mg/kg, Sinopharm Chemical Reagent Co., Ltd, Shanghai, China). The abdominal cavity was fully exposed to allow access into the thoracic cavity with an abdominal midline incision, avoiding lung or heart injury. The self-made rat lung lavage device (a 10-ml injector with 27-gauge needle) was inserted into the left ventricular apex of rats. The lavage was performed for approximately 2 min using PBS which was passed into the aorta from the left ventricle of heart and circulated throughout the body. When the pink lung tissues gradually turned pale and off-white, the left and right lung tissues were incised from the rats by rapid exposure of the trachea and lung. Portions of removed lung tissues were stored in liquid nitrogen, the rest of which was immersed in 4% paraformaldehyde and embedded with paraffin. Tissues were then sliced into successive sections (4-μm thick). These sections were preserved for later Hematoxylin–Eosin (HE) staining and immunohistochemistry. Terminal deoxynucleotidyl transferase (TdT) mediated dUTP-biotin nick end-labeling (TUNEL) staining was applied to detect the apoptotic rates of AECs.

### HE staining

Three lung tissue sections were randomly selected from each group. All sections were dewaxed with xylene and hydrated with ethanol. Sections were stained by Hematoxylin, and differentiated by hydrochloric acid-ethanol solution. Next, they were counterstained by Eosin, and finally dehydrated by ethanol. The samples were observed under light microscope after being dewaxed with xylene and sealed with neutral gum.

### Immunohistochemistry

The expression of PKR-like ER kinase (PERK) and CHOP proteins in lung tissues were measured by immunohistochemistry. Lung tissues were first sliced into sections, and then dewaxed with xylene and dehydrated by alcohol. The activity of endogenous peroxidase was blocked with the addition of 3% hydrogen peroxide. Then, the slices were transferred to 0.01 mol/l of citrate buffer solution (pH 6.0), and heated in a microwave oven to retrieve antigens for 20 min. PBS rinsing was conducted three times after natural cooling (5 min per rinse). After antigen retrieval, rabbit-anti-mouse PERK or CHOP monoclonal antibody (in the ratio of 1:500, Labvision Corporation, Fremont, California, U.S.A.), were added to the tissue sections and incubated at 37°C for 1 h. Tissue sections were then incubated at 37°C for another 30 min with the second antibody, biotinylated goat anti-rabbit IgG. Streptavidin-labeled horseradish peroxidase (S-A/HRP) was added to the tissues and was left to further incubate for 10–15 min at 37°C. Tissue sections were stained with diaminobenzidine (DAB) for 1–2 min, and washed with PBS three times (2 min per time). Tissue sections were counterstained by Hematoxylin for 1 min, dehydrated by alcohol, and sealed with neutral gum. The positive sections and PBS that replaced the primary antibody served as the positive control and negative control. After staining, the positive tissue sections appeared as brown or tawny-brown when observed under the microscope. The integrated optical density (IOD) values of tissue sections in each group were measured by Image-Pro Plus 6.0 software after tissue images were captured under an optical microscope (×400). Five views were randomly selected to determine the positive IOD values, and the mean IOD values were considered as the relative expressions of PERK and CHOP.

### TUNEL staining and determining apoptotic rates of AECs

The apoptotic rates of AECs in rats were detected using a TUNEL detection kit (Roche Ltd., Basel, Switzerland). The lung tissues of rats in all the three groups were fixed with 10% paraformaldehyde at room temperature for 30 min, and then incubated in an ice-bath with PBS containing 0.1% Triton X-100 for 2 min. After allowing to dry, 50 μl of the TUNEL reaction mixture (the ratio of enzyme solution and label solution was 1:9) was added to samples, and left to incubate in the wet box at 37°C for 60 min. Following a PBS wash, 50 μl of transforming agent was added to tissue samples, after which tissues were incubated in the wet box at 37°C for another 30 min. Tissue samples were washed with PBS, followed by coloration with 100 μl of DAB substrate solution. And 10 min later, tissues were observed under a light microscope. Yellow-brown granules observed in the nucleus of rats indicated TUNEL-positive cells. Three visual fields were randomly selected from each tissue section using a microscope, in which apoptotic AECs were counted and the mean apoptosis rate was calculated. Apoptotic rate was calculated as the number of apoptotic AECs divided by the number of total AECs.

### Western blotting

Proteins were extracted from lung tissues of rats in each group. The BCA assay (Beyotime Biotechnology Co., Shanghai, China) was performed to detect the total concentration of the proteins. SDS/PAGE (Beyotime Biotechnology Co., Shanghai, China) was performed to separate proteins. Separated proteins were transferred on to PVDF membrane, which was blocked with 5% skim milk and left on the shaker for 1 h at 37°C. Later, the proteins were treated with the primary antibodies against light chain 3 (LC3-II), Caspase-12, and β-actin (diluted in the ratio of 1:1000, Cell Signaling Technology, Beverly, MA, U.S.A.), rabbit-anti-rat p62 (ab56416, 1 μg/ml, Abcam, Cambridge, U.S.A.), rabbit-anti-rat Beclin-1 (ab62557s, 1 μg/ml, Abcam, Cambridge, U.S.A.), rabbit-anti-rat ATG5 (ab108327, 1 μg/ml, Abcam, Cambridge, U.S.A.), rabbit-anti-rat ATG7 (ab52472, Abcam, Cambridge, U.S.A., in the ratio of 1:100), and rabbit-anti-rat Caspase-3 (ab13847, Abcam, Cambridge, U.S.A., in the ratio of 1:500) at 4°C overnight. The membrane was then washed with TBS-Tween 20 (TBST). Protein samples were incubated for another 2 h with HRP-labeled goat anti-rabbit IgG (1:2500; Cell Signaling Technology, Beverly, MA, U.S.A.). After the membrane was washed, the proteins were developed with chemiluminescence reagent, and gray-scale value of protein bands were measured by ImageJ software. Formula: the relative expression of the target protein was calculated by dividing the gray-scale value of target band by the gray-scale value of internal reference band. Each experiment was repeated three times.

### Statistical analysis

All experimentally obtained data were analyzed by SPSS 21.0 statistical software (IBM Corp. Armonk, NY, U.S.A.). Measurement data were presented as a mean ± S.D., and comparison of data between two groups was conducted using a *t*test. All the statistics were bilaterally calculated with the significant test level of α =0.05. Values of *P*<0.05 were considered as statistically significant.

## Results

### General conditions and status of rats in the control, COPD, CQ intervention, and 3-MA intervention groups

The wounds of all the rats healed almost completely within a week after receiving intratracheal instillation of LPS or sterilized normal saline for the first time. When the rats underwent intratracheal instillation of LPS for the second time, rats in the control, CQ intervention, and 3-MA intervention groups recovered well. The healing rate of rats in the COPD group was slower than those after their first-time instillation. From the 15th to 28th day, rats in the control group retained a normal diet and appetite, sensitive response, and shiny skin, with a steady weight increase. In the COPD group, the rats exhibited a reduced diet intake, slow response, dry hair, and constant loss of the body weight. They also exhibited a rapid shallow and breathing in usual, and whoops under exposure to CS, accompanied with obvious paradoxical respiratory. The general conditions of rats in the 3-MA intervention and CQ intervention groups were worse than that in the control group but better than that in the COPD group.

### Evaluation of pulmonary function amongst the control, COPD, CQ intervention, and 3-MA intervention groups

Pulmonary function tests showed that the FEV_0.3_/FVC% and Cdyn were significantly lower and RI was significantly higher in the COPD group compared with the control group (all *P*<0.05). This indicates that the conditions and statuses of the rats (airflow obstruction and obstructive ventilatory dysfunction) were consistent with the changes in pulmonary function in the rat models of COPD. In the 3-MA intervention and CQ intervention groups, the FEV_0.3_/FVC% and Cdyn were significantly higher than those in the COPD group, while RI was lower than that in the COPD group (all *P*<0.05) (Table 1). No significant differences were found in the FEV_0.3_/FVC%, Cdyn, and RI between the control and COPD groups (all *P*>0.05).

**Table 1:** Comparison of pulmonary function parameters amongst the control, COPD, CQ intervention, and 3-MA intervention groups

Group	*n*	FEV_0.3_/FVC (%)	RI (ml/cm H_2_0)	Cydn (cm H_2_0/ml/S)
Control	14	82.18 ± 9.87	0.36 ± 0.04	0.35 ± 0.03
COPD	14	52.33 ± 8.60*	0.64 ± 0.06*	0.16 ± 0.02*
3-MA intervention	14	77.34 ± 9.34^#^	0.32 ± 0.04^#^	0.33 ± 0.03^#^
CQ intervention	14	78.32 ± 9.01^#^	0.35 ± 0.05^#^	0.31 ± 0.04^#^

*, *P*<0.05 compared with the control group; ^#^, *P*<0.05 compared with the COPD group.

### Histological changes in lung tissues belonged to rats in the control, COPD, CQ intervention and 3-MA intervention groups

Images of rat lung tissues stained with HE were shown as Figure 1. Integral bronchial epithelial cells (BECs) and AECs were visible in the control group. Thick bronchial wall, necrosis, and exfoliation of AECs, increase in number of infiltrated inflammatory cells in airway, pulmonary parenchyma and blood vessel, filmy alveolar wall, aneretic alveoli construction, partial alveolar fusion, pulmonary bullae and infiltration inflammatory cells in alveolar septum were seen in rats belonging to the COPD group. In the 3-MA intervention and CQ intervention groups, bronchial wall was slightly thickened, degeneration was observed in a few AECs, tracheal epithelium fell off, a lower amount of infiltrated inflammatory cells in airway and blood vessel compared with the COPD group were present, as well as a decrease in the fusion of pulmonary alveoli.

**Figure 1:** Histological observation of lung tissues of rats in the control, COPD, CQ intervention, and 3-MA intervention groups detected by HE staining (×200) The black arrow indicates inflammatory cells; the blue arrow shows the destroyed alveolus fused into pulmonary bullae.

### Decreased expressions of PERK and CHOP by suppressing autophagy in the 3-MA intervention and CQ intervention groups

The PERK positive expression dyed in the cytoplasm and the CHOP-positive expression dyed in the nucleus was visible in both BECs and AECs (Figure 2). The IOD values of PERK and CHOP of lung tissues belonging to the COPD group were significantly higher than those in the control group (both *P*<0.05). In the 3-MA intervention and CQ intervention groups, the IOD values of PERK and CHOP of lung tissues were significantly lower than those in the COPD group (both *P*<0.05). No significant difference was observed in the PERK and CHOP IOD values between the control and 3-MA groups (both *P*>0.05). These results indicated that the ERS was enhanced in the COPD group, which might be reduced by 3-MA intervention.

**Figure 2:** Comparison of IOD values of PERK and CHOP in lung tissue of rats amongst the control, COPD, CQ intervention, and 3-MA intervention groups *, *P*<0.05 compared with the control group; ^#^, *P*<0.05 compared with the COPD group.

### Low apoptosis rate of AECs in rats by inhibiting autophagy in the 3-MA intervention and CQ intervention groups

TUNEL staining demonstrated that the apoptotic rate of AECs in the COPD group were significantly higher than those in the control group (*P*<0.05). On the other hand, the apoptosis rate of AECs was markedly lower in the 3-MA intervention and CQ intervention groups compared with that in the COPD group (*P*<0.05). There was no significant difference in the apoptotic rates between the control and 3-MA intervention groups (*P*>0.05) (Figure 3).

**Figure 3:** The apoptotic rates of AECs in lung tissues of rats amongst the control, COPD, CQ intervention, and 3-MA intervention groups (**A**) Images of the apoptotic rates of AECs in lung tissues of rats amongst the control, COPD, CQ intervention, and 3-MA intervention groups detected by TUNEL staining (×400); (**B**) histogram of the apoptosis rate of AECs in rats amongst the control, COPD, CQ intervention, and 3-MA intervention groups; *, *P*<0.05 compared with the control group; ^#^, *P*<0.05 compared with the COPD group.

### Reduced expressions of autophagy-related proteins apoptosis-related proteins in rats with COPD

Western blotting was conducted to measure the expressions of apoptosis-related proteins in rats with COPD (Figure 4). Compared with the control group, the expression levels of LC3-II, Beclin-1, ATG5, ATG7, Caspase12, and Caspase-3 in lung tissues were significantly higher, but the expression of p62 expression was lower in the COPD group (both *P*<0.05). The 3-MA intervention and CQ intervention groups exhibited significant expressions of LC3-II, Beclin-1, ATG5, ATG7, Caspase12 and Caspase-3, and higher p62 expression in lung tissues compared with that of the COPD group (both *P*<0.05). No significant difference was found in the apoptotic related proteins expressions amongst the control, CQ intervention, and 3-MA intervention groups (both *P*>0.05).

**Figure 4:** Expression levels of autophagy-related proteins apoptosis-related proteins in rats with COPD amongst the control, COPD, CQ intervention, and 3-MA intervention groups (**A**) Histogram of the expression levels of autophagy-related proteins apoptosis-related proteins detected by Western blotting; (**B**) statistical analysis of gray values of expressions of autophagy-related proteins apoptosis-related proteins; *, *P*<0.05 compared with the control group; ^#^, *P*<0.05 compared with the COPD group.

## Discussion

In the present study, we investigated how the apoptosis of AECs induced by ERS in COPD rats as well as the protective effects of autophagy, can prove that the inhibition of autophagy itself might alleviate ERS-induced apoptosis of AECs in rat models of COPD. Autophagy is a natural cellular process during which protein and organelles are degraded in order to maintain cell viability and activity in response to nutrient limitation, and functions as a form cytoprotection and cell apoptosis [20,21]. Autophagy allows for the orderly degradation and recycling of cellular components to be used by other metabolic and cellular pathways [22].

Our study demonstrated that both 3-MA and CQ are beneficial in inhibiting the process of autophagy. 3-MA belongs to a group of phosphoinositide-3-kinase (PI3K) inhibitors, which have been widely used as autophagy inhibitors based on their inhibitory effects on class 3 PI3K activity, an essential component for the induction of autophagy [23]. Petiot et al. [24] helped to identify that the inhibitor 3-MA, is an early autophagy inhibitor, which could suppress the activity of type III of PI3K and the formation of autophagosome so as to inhibit autophagy. CQ can also act as an autophagy inhibitor that mainly inhibits the binding of autophagy to lysosomes to help prevent autophagosome degradation [25]. FEV_0.3_/FVC% and Cdyn decreased while the RI was increased in the COPD group compared with the control group. In the present study, the rat models of COPD were successfully established by CS inhalation. CS exposure leads to early neurogenic inflammation in the airways through stimulating sensory neurones causing CS-evoked diseases, such as asthma or COPD [26]. The signal transduction of unfolded protein response (UPR) is mediated by three transmembrane proteins which are known as PERK, ATF6, and IRE1 in the ER. While PERK, ATF6, and IRE1 could all help to initiate the apoptotic pathway and induce apoptosis when the ERS reaction is too strong or the duration is too long, when the damage is too extensive and exceeds the cell’s ability to instigate repair pathway. The corresponding mechanisms starts with the activation and transcription of CCAAT/CHOP, which leads to the activation of the C-jun/JNK signaling pathway and ultimately activating caspase pathways leading to production of Caspase12 [27]. Consistently, ERS could lead to increased cell apoptosis and autophagy in AECs by CS inhalation [28]. The decrease in the FEV_0.3_/FVC% ratio represents an inhibited pulmonary ventilation function, and the decreased Cdyn indicates low lung compliance with an increasing intrapleural pressure [29]. Airflow limitation is the end result of several main causes that contribute to COPD whereby an aggravated airway resistance is one of the most important causes [30]. Furthermore, a thick bronchial wall, the necrosis and exfoliation of AECs and pulmonary bulla were presented in rats that developed COPD. The thickening of the bronchial wall is typically found in patients with COPD, which may be negatively correlated with the degree of airflow obstruction [31]. Bullae can appear in healthy persons or patients with relatively rare hereditary diseases, but most bullae are associated with COPD and emphysema [32]. Interestingly, the FEV_0.3_/FVC% ratio and Cdyn significantly increased, whereby RI decreased in the 3-MA intervention and CQ intervention groups compared with that in the COPD group. Our results also indicated that the inhibition of autophagy can reduce bronchial wall thickening and pulmonary bullae in COPD rats. These results provided evidence that the inhibition of autophagy might improve pulmonary function in rats with COPD.

Sequentially, expressions of both PERK and CHOP in the COPD rats significantly increased. However PERK and CHOP expression levels both declined when autophagy was inhibited. The ERS is associated with specific proteins, such as PERK, CHOP, ATF4, GRP78, p-eIF2α, and Caspase12, whereby each of these proteins are closely associated with one another [33]. PERK is the major protein related to the attenuation of mRNA translation and is activated during ERS, inhibiting the influx of freshly synthesized proteins into the stressed ER compartment [34]. PERK phosphorylates eIF2α *in vitro*, and when overexpressed in cells, can lead to the attenuation of protein synthesis [35]. The transcription factor CHOP was first reported as a protein that was involved in ERS-induced apoptosis [36,37]. It is a transcription factor that can promote ERS-induced apoptosis by transcriptional induction, and it has been proved that its deficiency protected the cells from apoptosis induced by ERS [38]. CHOP expression is normally low under non-stressful conditions, but its expression markedly increased in response to ERS through IRE1, PERK and ATF6-dependent transcriptional induction. The results showed that inhibition of autophagy results in a reduced expression of PERK and CHOP in COPD rats. As a result, this may protect cells from ERS-induced apoptosis. In the present study, the expressions of autophagy protein LC3-II, Beclin-1, ATG5, ATG7, Caspase12, and Caspase-3 in lung tissues were significantly higher, but the p62 expression was lower in the 3-MA intervention and CQ intervention groups compared with the COPD group. Moreover, the apoptotic rates of AECs were remarkably suppressed in the 3-MA intervention and CQ intervention groups in comparison with the control group. LC3-II is a widely investigated protein marker of autophagy that binds to the autophagosome during autophagy [39]. Caspase12 is a protein that belongs to the family of enzymes called caspases which cleave substrates at C-terminal aspartic acid sequences. Caspases play a crucial role in apoptosis and inflammation. Caspase12 is a central molecule related to inflammasome activation and ERS-induced apoptosis, and may be activated by exposure to CS or some other components in CS [40]. Autophagy is up-regulated in epithelial cells of COPD patients, resulting in inflammation and emphysema in COPD [41,42]. Chen et al. [43] suggested that autophagy is a crucial and early response to CS, and ultimately promotes apoptosis in cells, thus potentially playing a vital role in the pathogenesis of COPD. Zhou et al. [44] also reported that autophagy is a critical response in the COPD pathogenesis that mediates pulmonary epithelial cell apoptosis as well as upstream and downstream signals of this pathway involve in CS-induced mucus production in mouse airways and human BECs. These results help support that the inhibition of autophagy may inhibit the ERS-induced apoptosis of AECs in COPD rats through regulating the apoptosis factor Caspase12.

In conclusion, our study mainly elucidated that the inhibition of autophagy improves pulmonary function and attenuates ERS-evoked AECs apoptosis in COPD rats exposed to CS. Therefore, the study supported that long-term 3-MA treatment might be a new therapeutic strategy for COPD. However, as a preliminary study, the underlying mechanism still needs to be validated by additional research with further attention paid to the regulation of cigarette smoking, inflammation, and reduction in ERS.

## Abbreviations

AEC: alveolar epithelial cell
BEC: bronchial epithelial cell
Cdyn: dynamic lung compliance
CHOP: CCAAT/enhancer-binding protein-homologous protein
COPD: chronic obstructive pulmonary disease
CQ: chloroquine
CS: cigarette smoke
DAB: diaminobenzidine
ER: endoplasmic reticulum
ERS: ER stress
FEV_0.3_/FVC%: forced expiratory volume in 0.3 s/forced vital capacity
HE: Hematoxylin–Eosin
HRP: horseradish peroxidase
IOD: integrated optical density
LC3-II: light chain 3
LPS: lipopolysaccharide
PERK: PKR-like ER kinase
PI3K: phosphoinositide-3-kinase
RI: inspiratory resistance
TUNEL: terminal deoxynucleotidyl transferase mediated dUTP-biotin nick end-labeling
3-MA: 3-methyladenine
